RETRACTED

# Data on the Impact of Epidemic on Nursing Staff's Mental Health in the Context of Wireless Network

**DOI:** 10.1155/2022/3413815

**Published:** 2022-04-07

**Authors:** Dan Guo, Yi Guo, YanJi Xing

**Affiliations:** ^1^Department of Operating Room, Central South University Xiangya School of Medicine Affiliated Haikou Hospital, Haikou 570208, Hainan, China; ^2^Department of Haikou Administrative Center Outpatient, Central South University Xiangya School of Medicine Affiliated Haikou Hospital, Haikou 570208, Hainan, China; ^3^Department of Health Medicine, Central South University Xiangya School of Medicine Affiliated Haikou Hospital, Haikou 570208, Hainan, China

## Abstract

The research was aimed to analyze the impact of epidemic pneumonia on nursing personnel's mental health under wireless network background and to improve the selection of random forest classification (RFC) algorithm parameters by the whale optimization algorithm (WOA). Besides, a total of 148 in-service nursing personnel were selected as the research objects, and 148 questionnaires were recycled effectively. The collected data were analyzed by the improved RFC algorithm. In addition, the research investigated the impacts of demographic factors on nursing personnel's mental health by the one-way variance method. The results demonstrated that the accuracy of the improved algorithm in training samples and test samples reached 83.3% and 81.6%, respectively, both of which were obviously higher than those of support vector machine (SVM) (80.1% and 79.3%, respectively) and back-propagation neural network (BPNN) (78.23% and 77.9%, respectively), and the differences showed statistical meanings (*P* < 0.05). The *Patient Health Questionnaire-9* (PHQ-9) showed that the depression levels of 9.46% of the included personnel were above moderate. The *Generalized Anxiety Disorder* (GAD-7) demonstrated that the anxiety levels of 3.38% of the included personnel were above moderate. The insomnia severity index (ISI) indicated that the insomnia levels of 3.38% of the included personnel were above moderate. The average score of male personnel (3.65) was obviously lower than that of female personnel (3.71). Besides, the average scale score of married personnel (3.78) was significantly higher than that of unmarried personnel (3.65). The average scale scores of personnel with bachelor's (3.66) and master's degrees (3.62) were obviously lower than those of personnel with junior college (3.77) and technical secondary school (3.75) diplomas. The average scale score of personnel with over 5-year work experience (3.68) was significantly lower than that of personnel working for less than five years (3.72). The average scale score of personnel with experience in responding to public emergencies (3.65) was obviously lower than that of personnel without related experience (3.74). The differences all showed statistical meaning (*P* < 0.05). The results of this research revealed that the accuracy of the improved RFC algorithm was remarkably higher than that of the SVM and BPNN algorithms. Furthermore, many nursing personnel suffered from mental diseases at different levels with the impact of the epidemic. Gender, marital status, education level, and experience in responding to public emergencies were the main factors affecting nursing personnel's mental health.

RETRACTED

## 1. Introduction

Health emergencies refer to sudden serious infectious diseases that cause (may cause) damage to the health of the vast majority of people, as well as mass diseases of unknown cause [1]. The outbreak of pneumonia in December 2019 was a type of health emergency, and this outbreak was lethal. Due to the suddenness of the disease, the relevant departments did not formulate effective solutions, resulting in a surge in the number of infections at home and abroad in a short period of time [2, 3]. According to relevant investigations and studies, the incubation period is generally 3 to 7 days, and some can even incubate for 14 days. The clinical presentation of this epidemic is similar to that of the common cold, with some atypical symptoms, including dry cough and fever [4–7]. Advances in wireless networking technology have allowed researchers to rapidly collect data on global infections [8, 9]. According to big data statistics, as of May 2021, there had been more than 140 million confirmed cases worldwide, with a case fatality rate of about 2.1%, causing serious harm to the country and its people [10, 11]. Mental health refers to the promotion and maintenance of people's psychological states through positive and beneficial measures to adapt to changes in the natural and social environment [12]. However, people's mental health has been greatly harmed by the epidemic. As front-line personnel in the fight against the pneumonia epidemic, medical staff shoulder the great responsibility of curing diseases and promoting health. They were hurt the most. Therefore, research on the psychological and stress responses of medical staff has become a hotspot [13, 14].

Traditional mental health survey methods are passive and inaccurate. Patients' mental health states can be determined only by the active consultation with psychologists and the implementation of professional detection [15]. Psychologists diagnose and treat patients' diseases mainly by communicating with patients and giving out questionnaires, which is greatly affected by the subjective factors of doctors, and the diagnosis and treatment based on this method are inaccurate [16]. With the development of medical treatment, science, and technology, the active description is not the only method of diagnosing patients' mental states. Some scholars detect brain waves, heart rate, and electrical signals by apparatuses designed by wireless networks and artificial intelligence (AI) technology to reflect the current mental state of patients. As result, there are the intersection and combination between AI technology and psychology [17]. With the background of big data, AI promotes the rapid development of Internet technology as well as generates massive data. The extraction of useful information from these massive data is a major difficulty in the current development of Internet technology [18]. The decision tree (DT) algorithm is a kind of typical single classifier among many classification algorithms, which is applied in a great many fields [19]. However, the issues needed to be tackled by classifiers have become gradually complex with the development of human society. Hence, DT algorithm-based classifiers are significantly limited [20]. Random forest classification (RFC) is a kind of common combined classification method, which adopts DT as basic classifiers, and it is usually applied in mental diagnostic classification [21]. RFC is pervasive, and the excellent anti-noise capacity as well as the tolerance of abnormal values are advanced in data mining. Nevertheless, the classification results are affected by the artificial setting of the RFC algorithm parameters. Therefore, the methods of reducing the generalization errors of the RFC algorithm need to be improved [22, 23]. The whale optimization algorithm (WOA) is a new nature-inspired metaheuristic optimization algorithm that simulates the social behaviors of humpback whales and introduces a bubble net hunting strategy. The algorithm has a simple structure, few parameters, strong search capability, and is easy to implement. However, the research and application of WOA is still in its initial stage, and the algorithm itself still has the disadvantages of low solution accuracy, slow convergence speed, and is easy to fall into local optimum. The BP neural network is the most basic neural network, whose output is propagated forward and the error is propagated backward, and the BPNN is widely used in classification and regression problems due to its strong nonlinear mapping ability and high self-learning and adaptive capabilities. BP neural networks can automatically extract the “reasonable rules” between the output and the output data and adaptively memorize the learning content in the network weights. BP neural networks have a high degree of self-learning and self-adaptive ability, and it is difficult to solve the contradiction between the size of the application problem and the size of the network, which involves the relationship between the possibility of network capacity and feasibility, i.e., the problem of learning complexity.

RETRACTED

To sum up, the research was based on the random forest (RF) algorithm, which was improved and applied in data analysis to investigate the impact of the epidemic on nursing personnel's mental health under the background of wireless network. In addition, nursing personnel's mental health states were studied and analyzed by survey to offer an effective decision analysis to nursing personnel's mental health and clinical work.

## 2. Materials and Methods

### 2.1. Research Objects

A total of 148 in-service nurses working at Central South University Xiangya School of Medicine Affiliated Haikou Hospital from May 2020 to August 2020 were selected as the research objects in the research, which included 42 male cases and 106 female cases aged between 19 and 54. Their average age was 34.23. Besides, the general data on the included nurses were collected. The research objects were included in the research based on the following standards: the included cases must be the front-line nurses with more than 1-year work experience, and they should be equal to or over 18 years old. The nurses were excluded by the research based on the following standards: those on further training or internship were excluded from the research, and those with previous neurasthenia and mental trauma were also excluded from the research. The implementation of this research has been approved by the Central South University Xiangya School of Medicine Affiliated Haikou Hospital Medical Ethics Committee, and all research objects have been informed about the research and volunteered to engage in the research.

### 2.2. Survey Tools

Questionnaires mainly consisted of the following several types of data (Table 1). Including the first one was the general data of the research objects, *Patient Health Questionnaire-9* (PHQ-9), *Generalized Anxiety Disorder* (GAD-7), and Insomnia Severity Index (ISI).

### 2.3. Survey Methods

The online questionnaire method was adopted in the research. All questionnaires were shared in the form of quick response (QR) code onto the electronic communication devices of 148 nursing personnel through WeChat. All the survey items designed in the research were compulsory. To avoid repeat answers, each case was allowed to answer each item once only, and relevant staff were arranged to answer questions raised by confused nursing personnel. In the research, a total of 148 questionnaires were handed out, and 148 valid questionnaires were recycled with the recycling efficiency reaching 100%.

RETRACTED

### 2.4. AI Algorithm and Its Improvement

The RF algorithm was introduced as follows: DT consisted of nodes and directed edges. Nodes contained root nodes, internal nodes, and leaf nodes (root nodes were the assembly of the whole training data, internal nodes referred to a certain feature or property, and leaf nodes represented a certain category). Each node could be split into DT, and leaf nodes could be viewed as the data sets containing classification labels. As a result, DT could be regarded as the exploration of the path to the classification. However, DT could not process continuous variables effectively, and the classification rules were complex. In addition, overfitting occurred if there were few training data. The RFC algorithm was a classification algorithm based on the combination of multiple DT, and it was a kind of typical classifier among ensemble learning algorithms. Ensemble learning refers to the assembly of excellent performances to solve complex tasks by adopting different combined algorithms. The structure of classifiers consisted of *n* corresponding functions generated by *n* classifiers, and these functions were combined with others according to certain rules to generate a combined classifier. The RFC algorithm was the combined form of multiple classifications (Figure 1).

It was assumed that *α* referred to random parameter vectors, *α*_1_ was the corresponding vector of *α* in the DT *T*, m represented test samples, and lead nodes were expressed as *e*(*m*, *α*), and then the RFC algorithm was further discussed in this study.

Bootstrap resampling was adopted to generate *x* training sets, which were marked with *α*_1_, *α*_2_, *α*_3_,…, *α*_*x*_, respectively. In each training set, the corresponding DT was generated and marked as {*T*(*m*, *α*_1_)}, {*T*(*m*, *α*_2_)}, {*T*(*m*, *α*_3_),…, {*T*(*m*, *α*_*x*_)}, respectively. If features had P dimensions, *p* features were selected randomly from P dimensions as the classification feature set of the node. The nodes were classified by the classification method with the best effect among *p* features to make each DT grow to the maximum size. F was set to be test samples, and the trained DT were adopted in tests to generate the corresponding categories, including {*T*(*f*, *α*_1_)}, {*T*(*f*, *α*_2_)}, {*T*(*f*, *α*_3_)} … {*T*(*f*, *α*_*x*_)}. The voting method was utilized to set the category with the most output in *x* DT as the category of the test set sample F.

The improvement of the RFC algorithm was as follows: the results predicted by RFC were susceptible to the number of DT in forests, feature subsets, and leaf nodes, which reduced the classification accuracy. To reduce the forecast errors by the RFC algorithm, a whale optimization algorithm (WOA) [24] was introduced in the research to improve the RFC algorithm. The classification accuracy A was selected as fitness function, which was expressed by (1) as follows:

(1) $$\begin{array}{c} A=\frac{R}{T}\times 100\%\#. \end{array}$$

In (1), *R* refers to the number of samples correctly classified, and *T* denotes the total number of samples. The process of the optimized RFC algorithm was explained as follows: the evaluation indexes of nursing personnel's mental health were set as the initial data, and then the training set (M) and the test set (F) of the RFC algorithm were obtained. After that, data were normalized as shown in (2) as follows:

(2) $$\begin{array}{c} m^{1}=q+\left(\frac{m-m_{min}}{m_{max}-m_{min}}\right)\times \left(w-q\right). \end{array}$$

In equation (2), *m*^*1*^ represents the training set data after normalization, *m* refers to the initial data, *m*_min_ denotes the minimum value of the initial data, *m*_max_ means the maximum value of the initial data, *q* represents for the minimum value after normalization, and *w* refers to the maximum value after normalization. In the research, *q* was assigned with the value −1, and *w* was assigned with the value 1.

RETRACTED

The colony size and the number of iterations were set to be Y and *s*, respectively. Besides, the position of whales was randomly initialized as *M*_*i*_(*i*=1,2,3,…, *n*). The number of DT, feature subsets, and the number of leaf node samples were also initialized. Based on (1), the fitness of each individual in whales was obtained. The best number of whales *M*^*1*^ were selected and saved. In addition, the best fitness of individuals in whales and the corresponding spatial position were output to obtain the parameters of the optimal colony, including the number of DT, feature subsets, and leaf nodes (Figure 2). In addition, a 17 : 3 ratio of test data to training data was used in this study.

### 2.5. Observation Indexes

Figure 3 demonstrates the evaluation of the classification effects of two types of classifier algorithms, including back-propagation neural network (BPNN) [25] and support vector machine (SVM) [26] by confusion matrix. BP neural networks are the most basic neural networks, with forward propagation of the output and backward propagation of the error. It imitates the activation and transmission processes of human neurons. Taking the three-layer neural network as an example, the BP neural network contains three layers of structure: an input layer, a hidden layer, and an output layer. The input layer receives data, the output layer outputs data, and the neurons in the previous layer are connected to the neurons in the next layer, collecting information from the neurons in the previous layer and passing the values to the next layer after “activation.” BPNN has nonlinear mapping capability, self-learning and self-adaptive capability, generalization capability, and fault tolerance.

RETRACTED

*TP* denotes positive real values, *TN* refers to negative real values, *FP* represents positive forecast values, and *FN* represents for negative forecast values. The accuracy was expressed by (3) as follows:

(3) $$\begin{array}{c} accuracy=\frac{TP+TN}{TP+TN+FP+FN}. \end{array}$$

### 2.6. Statistical Analysis

In the research, Statistical Product and Service Solutions (SPSS) 19.0 statistical software was adopted to analyze and process data. The measurement data were expressed by the mean ± deviation $\left(\bar{X}\pm S\right)$, and the enumeration data were denoted by percentage mark (%). Besides, one-way variance analysis was adopted in pairwise comparison, and *P* < 0.05 indicated that the differences showed statistical meanings.

## 3. Results

### 3.1. Experimental Test

To test the application effects of the improved RFC algorithm (n-RFC), nurse mental health questionnaires from 2018 to 2019 at Central South University Xiangya School of Medicine Affiliated Haikou Hospital were retrospectively analyzed in the research, and the survey results were included as the research objects. Besides, 85% of data were selected randomly from the sample data as the training data, and the rest were set as the test data. In addition, BPNN and SVM classifiers were compared, and the forecast accuracy of the results (three health dimensions including anxiety, depression, and fear) by three types of algorithms was compared based on expert judgment (Figure 4).

According to the abovementioned three results, the accuracy of three algorithms in training samples and test samples could be calculated. The accuracy of the n-RFC algorithm, SVM algorithm, and BPNN algorithm in training samples was 83.3%, 80.1%, and 78.23%, respectively, while those in test samples were 81.6%, 79.3%, and 77.9%, respectively (Figure 5). Obviously, the accuracy of the n-RFC algorithm in training samples was significantly higher than that of the SVM and BPNN algorithms, and the differences showed statistical meaning (*P* < 0.05).

### 3.2. Basic Data Statistics

A total of 148 research objects were included in the research, and 148 valid questionnaires were obtained, including 42 and 106 statistical results of data on males (28.37%) and females (71.63%), respectively. Most of the included research objects were aged between 27 and 45 (50.67%), and the proportion of the research objects with bachelor's degrees in the research objects at different education levels was the highest (52.03%) (Table 2).

RETRACTED

### 3.3. Statistics Results of Each Scales

#### 3.3.1. PHQ-9

Figure 6 demonstrates the survey results of depression of 148 nursing personnel in the past 2 weeks. Among depression-related symptoms in PHQ-9, most of the cases suffered from A (pleasure loss), C (sleep disorder), D (energy lack), E (eating disorder), and G (difficulty in concentration) for more than half the time in the past 2 weeks, and the proportion of the incidence of the above 5 symptoms in that of all symptoms in the past 2 weeks reached 6.08%, 8.78%, 6.76%, 6.76%, and 8.1%, respectively.

#### 3.3.2. GAD-7

Figure 7 shows the survey results of the depression of 148 nursing personnel in the past 2 weeks. Among depression-related symptoms in GAD-7, A2 (dysphoria), B2 (failure to control concern), C2 (energy lack), and F2 (fidget) occurred over half the time in the past 2 weeks among most of the cases, and the proportion of the incidence of the above 4 symptoms in that of all symptoms in the past 2 weeks amounted to 4.05%, 4.05%, 4.73%, and 3.38%, respectively.

#### 3.3.3. ISI

Figure 8 reveals the survey results of the sleep status of 148 nursing personnel in the past 2 weeks. Among the insomnia-related symptoms in ISI, A3 (difficulty in falling asleep), B3 (difficulty in maintaining sleep), C3 (early awakening), D3 (satisfaction with sleep), E3 (impacts on daily activities), F3 (impacts on living quality), and G3 (worry/pain) manifested at moderate levels among 9.23%, 8.66%, 7.25%, 22.61%, 8.02%, 5.01%, and 7.57% of the included research objects in the past 2 weeks. Among all the symptoms manifesting at severe and extremely severe levels, the proportions of dissatisfaction with sleep among the included research objects were the highest, reaching 7.43% and 2.03%, respectively.

### 3.4. Overview of Anxiety, Depression, and Insomnia

Based on the abovementioned statistical results, the data were analyzed by the n-RFC algorithm in the research, which is shown in Figure 9. According to the statistical results, the average scores of 148 nursing personnel by PHQ-9, GAD-7, and ISI were 4.01 ± 4.09, 4.12 ± 4.27, and 2.87 ± 3.08, respectively. According to PHQ-9, the depression levels of 14 cases were above moderate; GAD-7 revealed that the anxiety levels of 5 cases were above moderate; and ISI showed that the insomnia levels of 5 cases were above moderate. To reflect the grading of different levels in different scales more intuitively, the proportions of different levels were presented (Figure 9(c)).

RETRACTED

### 3.5. Single Factor Analysis of Factors Affecting Nursing Personnel's Mental Health

Figure 10 demonstrates the single factor analysis of the factors affecting nursing personnel's mental health. According to the results, the average score of males (3.65) was lower than that of females (3.71), the average score of scales of married nursing personnel (3.78) was obviously higher than that of the unmarried (3.65), and the average scores of nursing personnel with bachelor's (3.66) and master's (3.62) degree were obviously lower than those of nursing personnel with junior college diploma (3.77) and technical secondary school diploma (3.75). Besides, the average score of nursing personnel with more than 5-year work experience (3.68) was significantly lower than that of those working for less than 5 years (3.72). The average score of nursing personnel with experience in responding to public emergencies (3.65) was obviously lower than that of those without related experience (3.74), and the differences all demonstrated statistical meaning (*P* < 0.05).

## 4. Discussion

The pneumonia outbreak that occurred in 2019 is an acute respiratory disease that is highly contagious. This is another health emergency following the 2003 SARS and the 2009 infection of the A hemagglutinin 1 neuraminidase 1 (H1N1) population [27]. It not only directly threatens physical life and health but also greatly affects people's mental health [28]. As the front-line team in the fight against the epidemic, the mental health of nursing staff has received much attention. Therefore, the study used the RFC algorithm to analyze the impact on the mental health of nursing staff in the context of wireless networks [29]. Traditional RFC algorithms were susceptible to the number of DT, feature subsets, and leaf nodes, which resulted in significant errors in forecast results [30]. Weng et al. [31] improved the forecast accuracy of cardiovascular risks by adopting the RFC algorithm in wireless network technology and machine learning. In this research, the WOA algorithm was introduced, and the selection of RFC algorithm parameters by the self-adaptability of the WOA algorithm. To verify the forecast performance of the improved algorithms, SVM and BPNN algorithms were introduced in the research. Besides, the data on nurse mental health questionnaires from 2018 to 2019 were included as the research objects to analyze the accuracy of three types of algorithms. The results demonstrated that the scores of three health dimensions, including anxiety, depression, and fear, were 0.56, 0.34, and 0.42, respectively, according to the experts' analysis. In contrast, the forecast scores of anxiety, depression, and fear by the n-RFC algorithm were 0.54, 0.32, and 0.46, respectively. Compared with those by SVM and BPNN, the forecast scores generated by n-RFC algorithm were more similar to the results of expert analysis. In addition, expert analysis results were set as the standard for the comparison of the forecast accuracy of the n-RFC, SVM, and BPNN algorithms. The results showed that the accuracy of the n-RFC algorithm in training and test samples was 83.3% and 81.6%, respectively, which was significantly higher than those of the SVM algorithm (80.1% and 79.3%) and the BPNN algorithm (78.23% and 77.9%), and the differences demonstrated statistical meaning (*P* < 0.05). The above results revealed that the improved algorithm was more accurate and had potential in data analysis to some degree.

RETRACTED

In the research, a total of 148 in-service nursing personnel were included as the research objects, and 148 questionnaires were recycled effectively. To collect more specific data, 3 scales were introduced in the questionnaire designed in the research in total. The PHQ-9 scale mainly reflected the degree of depression, the GAD-7 scale mainly reflected the degree of anxiety, and the ISI scale mainly reflected insomnia. The results of the research showed that most included cases suffered from pleasure loss, sleep disorder, energy lack, eating disorder, and difficulty in concentration over half the time of the past 2 weeks among depression-related symptoms in PHQ-9, and the proportions of the above cases in all cases with each symptom were 6.08%, 8.78%, 6.76%, 6.76%, and 8.1%, respectively. Among depression-related symptoms in GAD-7, most of the cases suffered from dysphoria, failure to control concern, energy lack, and fidgeting over half the time in the past 2 weeks, and the proportions of the above cases in all cases with each symptom were 4.05%, 4.05%, 4.73%, and 3.38%, respectively. Among the insomnia-related symptoms in ISI, most of the cases suffered from difficulty in falling asleep, difficulty in maintaining sleep, early awakening, dissatisfaction with sleep, impacts on daily activities, impacts on living quality, and worry/pain at moderate levels in the past 2 weeks, and the proportions of the above cases in all cases with different levels of each case were 9.23%, 8.66%, 7.25%, 22.61%, 8.02%, 5.01%, and 7.57%, respectively. In addition, the n-RFC algorithm was adopted to analyze the collected data in the research, which revealed that the average scores of the PHQ-9, GAD-7, and ISI scales of 148 nurses were 4.01 ± 4.09, 4.12 ± 4.27, and 2.87 ± 3.08, respectively. According to PHQ-9, the depression levels of 14 cases (9.46%) were above moderate. GAD-7 indicated that the anxiety levels of 5 cases (3.38%) were above moderate, and the insomnia levels of 5 cases (3.38%) were above moderate. The epidemic broke out suddenly and was extremely contagious. The constant growth of the infected population and clinical infected cases caused certain mental pressure for medical care personnel, and few of them ever got involved in large-scale sudden sanitation events like this. With the lack of related solutions, they often felt anxious and depressed. According to the study conducted by Pollock et al. [32], antistress ability could be enhanced by workplace interventions, interventions to support basic and daily needs, mental support interventions, and drug interventions during the epidemic. With the current advanced wireless network technology, people can know about real-time epidemic development by intelligent devices. Regular epidemic prevention training and mental training for nursing personnel need to be provided. Besides, nursing personnel's mental pressure could be alleviated by mental preparation for emergencies at any time.

RETRACTED

In addition, the factors that affected nursing personnel's mental health were analyzed in the research, which showed that the differences of the impacts of age on nursing personnel's mental health demonstrated no statistical meaning (*P* > 0.05), and the average score of a male (3.65) was obviously lower than that of a female.

The results of the research also indicated that the scale average score of married nursing personnel (3.78) was significantly higher than that of unmarried. The average scores of nursing personnel with bachelor's (3.66) or master's (3.62) degree were obviously lower than those of nursing personnel with junior college or technical secondary school diplomas. Besides, the average scores of nursing personnel with more than 5-year work experience (3.68) were obviously lower than those of nursing personnel with less than 5-year work experience. The average score of nursing personnel with experience in responding to public emergencies (3.65) was significantly lower than that of nursing personnel without related experience, and the differences showed statistical meaning (*P* < 0.05). The differences resulted mainly from females' sensitivity compared with males. Besides, the antistress ability of females was significantly poorer than that of males because of body hormones. Because married nursing personnel often needed to care for their families and spouses, they felt more stressed compared with unmarried nursing personnel. The professional and mental qualities of nursing personnel with higher education levels were both higher than those of nursing personnel with lower education levels. Besides, the mental enduring capacity of nursing personnel with more working years was stronger than that of nursing personnel with fewer working years. According to the survey and study conducted by Spoorthy et al. [33], some sociodemographic variables were related to the pressure on medical care personnel, anxiety, depression, and insomnia, such as gender, occupation, age, workplace, and department. Furthermore, some mental variables, such as social support and self-efficacy, were also related to the pressure on medical care personnel, anxiety, depression, and insomnia. In addition, the nursing personnel with experience in responding to public emergencies showed less anxiety and fear than those without related experience in coping with them. Therefore, nursing staff should be encouraged to share their clinical nursing experience in responding to the pneumonia epidemic and praise the value of their experience in fighting the epidemic with positive actions.

RETRACTED

## 5. Conclusion

In the research, the selection of the RFC algorithm parameters was improved by the WOA algorithm. Besides, a total of 148 in-service nursing personnel were included as the research objects, and 148 questionnaires were recycled effectively. The collected data were analyzed by the improved RFC algorithm. In addition, the single factor analysis method was adopted to investigate the impacts of demographic factors on nursing personnel's mental health in the research. The results demonstrated that the accuracy of the improved RFC algorithm was obviously higher than that of the SVM and BPNN algorithms. Under the impact of the epidemic, many nursing personnel suffered from mental diseases at different levels. Gender, marital status, education levels, and experience in responding to sudden sanitation events were the main factors affecting nursing personnel's mental health. Nevertheless, the sample size was small compared with the global epidemic. Furthermore, the results of the research were incomprehensive, such as the lack of research results of the factors affecting nursing personnel's mental health. In future research, the sample size needs to be enlarged, and the impact of job factors on mental health should be increased. In general, the research offered data support to the elimination of the adverse impact of the epidemic on medical care personnel's mental health.

## Figures and Tables

**Figure 1:** Classifier composition diagram.

**Figure 2:** Optimized RFC algorithm framework after introduction of WOA algorithm.

**Figure 3:** Confusion matrix diagram.

RETRACTED

**Figure 4:** Comparison results of mental health dimensions and algorithms based on nurse mental health questionnaires from 2018 to 2019 as research objects. (a) The health dimensions of depression. (b) The health dimensions of depression. (c) The health dimensions of fear.

**Figure 5:** Comparison of the accuracy of n-RFC, SVM, and BPNN algorithms in training samples and test samples based on nurse mental health questionnaires from 2018 to 2019 as research objects. Note: ^*∗*^indicates that the comparison with the accuracy of the n-RFC algorithm showed statistical meaning (*P* < 0.05).

**Figure 6:** Statistics results of 148 nursing personnel in the past 2 weeks by PHQ-9 questionnaires. A refers to pleasure loss, B indicates depression, C represents for sleep disorder, D represents energy lack, E denotes to eating disorder, F means low self-evaluation, G refers to difficulty in concentration, H represents dysphoria, and I means negative ideas.

**Figure 7:** Statistics results of 148 nursing personnel in the past 2 weeks by GAD-7 questionnaires. A2 refers to dysphoria, B2 represents failure to control concern, C2 denotes the concern about this kind of thing, D2 means tension without relaxation, E2 represents for fidget, F2 represents irritability, and G2 indicates the fear that something bad would happen.

**Figure 8:** Statistics results of 148 nursing personnel in the past 2 weeks by ISI questionnaires. A3 refers to difficulty in falling asleep, B3 denotes difficulty in maintaining sleep, C3 represents early awakening, D3 denotes for dissatisfaction with sleep, E3 indicates impacts on daily activities, F3 means impacts on living quality, and G3 refers to worry/pain.

**Figure 9:** n-RFC data analysis diagram of the general results of 148 nursing personnel in the past 2 weeks by PHQ-9, GAD-7, and ISI, respectively. (a) The average scores of three scales, and error bars denoted the average score standard deviation of each scale of 148 nursing personnel. (b) The population statistics. (c) The general proportion of each level.

**Figure 10:** Single factor analysis of factors affecting 148 nursing personnel's mental health. (a) Gender and age groups. (b) Marital status and education levels. (c) Working years and experience in responding to public emergencies. Note: ^*∗*^indicated that the comparison with the average scores of other factors in the same group showed statistical meaning (*P* < 0.05).

**Table 1:** Specific items of questionnaire.

Questionnaire item type	Explanations
General data statistics	The collected general data on the research objects included gender, age, marital status, education level, working years, and experience in responding to public emergencies.

PHQ-9	The survey scale consisted of 9 items, including pleasure loss, depression, sleep disorder, energy lack, eating disorder, low self-evaluation, difficulty in concentration, dysphoria, and negative ideas. Each item was scored between 0 and 3. 0 referred to no occurrence, 1 represented an occasional occurrence, 2 meant that more than half of the above symptoms occurred, and 3 indicated an everyday occurrence. The total score between 0 and 4 stood for no depression, that between 5 and 9 referred to mild depression, that between 10 and 14 was moderate depression, and that over 15 denoted severe depression.

GAD-7	The survey scale consisted of 7 items, including dysphoria, control concern, concern about this kind of thing, tension without relaxation, fidget, irritability, and the fear that something bad would happen. Each item was scored between 0 and 3.0 referred to no occurrence, 1 represented an occasional occurrence, 2 meant that more than half of the above symptoms occurred, and 3 indicated an everyday occurrence. The total score between 0 and 4 represented no depression, that between 5 and 9 meant mild depression, that between 10 and 14 referred to moderate depression, and that over 15 denoted severe depression.

ISI	The survey scale consisted of 7 items, including difficulty in falling asleep, difficulty in maintaining sleep, early weakening, dissatisfaction with sleep, impacts on daily activities, impacts on living quality, and worry/pain. The full score for each item was 4. 0 referred to no insomnia, 1 represented mild insomnia, 2 denoted moderate insomnia, 3 stood for severe insomnia, and 4 meant extremely severe insomnia. The total score between 0 and 7 represented no insomnia, that between 8 and 14 referred to mild insomnia, that between 15 and 21 denoted moderate insomnia, and that between 22 and 28 indicated severe insomnia.

RETRACTED

**Table 2:** Basic data statistics of nursing personnel.

Items		Number of cases	Proportion (%)
Gender	Male	42	28.37
	Female	106	71.63

Age group (years)	19∼26	45	30.41
	27∼45	75	50.67
	46∼54	28	18.92

Marital status	Married	78	52.7
	Unmarried	70	47.3

Education level	Technical secondary school diploma	6	4.05
	Junior college diploma	62	41.89
	Bachelor's degree	77	52.03
	Master's degree	3	2.03

Working years	More than 5 years	62	41.89
	Less than 5 years	86	58.11

Experience in responding to public emergencies	Experienced	71	47.97
	No experience	77	52.03

## Data Availability

The data used to support the findings of this study are included within the article.
